# Spatial-Temporal Change Trend Analysis of Second-Hand House Price in Hefei Based on Spatial Network

**DOI:** 10.1155/2022/6848038

**Published:** 2022-05-23

**Authors:** Zheng Yin, Rui Sun, Yuqing Bi

**Affiliations:** School of Economics and Management, Anhui Jianzhu University, Hefei, Anhui, China

## Abstract

Spatial Markov chain can effectively explore the spatial evolution trend of housing price under the influence of lag factor. This paper uses spatial autocorrelation and spatial Markov to study 353 second-hand houses in Hefei. The results show that (1) the housing price of Hefei urban area presents a situation of “two points and one side,” the high housing price is concentrated in the south and southwest of the urban area, and the price level gradually weakens from south to north, and the housing development shows a north-south differentiation. (2) There is a significant spatial autocorrelation between second-hand housing prices in Hefei. The “high-high” residential price clusters are mainly distributed in Shushan District and Binhu New Area, while the “low-low” residential price clusters are mostly in Yaohai district and its surrounding areas. The number of “low-high” agglomeration and “high-low” agglomeration is small, and the degree of change is not big. (3) Under the influence of different neighborhood environments, the housing prices in urban Area of Hefei show club convergence overall. At the same time, under the short-term influence of the policy, the housing prices of low level and middle and low level are promoted in the same neighborhood environment, while the housing prices of high level and middle and high level are negatively affected.

## 1. Introduction

Housing is a major issue concerning people's livelihood, affecting the basic livelihood of millions of families. With the continuous improvement of economic life, the demand of house buyers is getting higher and higher. However, in order to meet the needs of residents, real estate developers actively launch differentiated housing products, so as to broaden the range of housing options for residents, but also produce some negative effects: urban living space misallocation, obvious spatial differentiation, housing prices, housing prices causing “speculation,” eventually leading to excessive real estate investment, forming the “bubble economy,” but really needing just to be difficult to meet the residents of housing, affecting the well-being of the people, which is not conducive to social stability and harmonious [1].

Hefei is a large city with a population of 10 million. Compared with 2010, its permanent population increased by 1.91 million, and the proportion of urban population increased by 20 percentage points [2]. Rapid urbanization and population agglomeration bring about increased demand and supply pressure for housing. The exuberance of demand and the relative reduction of supply cause the distortion of the market and the relationship between supply and demand. Under the combined action of multiple factors, such as the rise of land price and the influx of investors into the market, the real estate market in Hefei appears irrational overheating and fails to meet the demands of consumers with real rigid demand for housing [3]. In order to promote the steady and healthy development of Hefei real estate market, Hefei city issued new real estate policies in early April 2021, which began to strictly manage the land market and real estate market, strictly regulate the price of commercial housing, and severely crack down on all kinds of real estate market disorder.

Taking 353 second-hand residential houses in Hefei as the research object, this paper analyzes the spatial distribution difference of housing prices in different regions by means of mathematical statistics and spatial analysis (see Figure 1) and explores the rule of housing price type transformation under the influence of policies. It aims to promote the benign development of Hefei housing market, solve the real estate market disorder and supply and demand contradiction, and provide reference for Hefei municipal government and planning departments to formulate regional housing price regulation policies and public facilities planning.

## 2. Literature Review

As immovable property, a house has not only the basic property of living, but also high investment value. Different lots of real estate, the future appreciation space has also different size, because its high purchase cost limits the consumer group's choice range. Therefore, the change trend of housing price is one of the hot issues with the highest social attention. In recent years, many domestic scholars have introduced spatial data to study its spatial correlation and structure based on the use of traditional econometric models. The spatial distribution of urban residential prices has been studied from a spatially macroscopic perspective, and the patterns and causes of residential price changes in space have been quantified and analyzed by constructing a mathematical analysis model.

Kriging interpolation method can study the spatial differentiation of housing prices and the spatial distribution characteristics and evolution rules of housing prices, and explore the evolution trend of the outward diffusion of regional housing spatial development in recent years [4–7]. Compared with other interpolation methods, Kriging method not only considers spatial correlation, but also results are more reliable when there are more data points [4]. Kriging is an accurate local interpolation technique, which takes into account the spatial orientation of sample points and the spatial position relationship with unknown sample points [5].

Moran's I index is often used as a tool to analyze the spatial correlation and heterogeneity of housing prices, and reflects the spatial agglomeration and dispersion characteristics of housing through significance [8–13]. Global spatial autocorrelation is an assessment of the degree of spatial autocorrelation, which reflects the overall trend of spatial correlation of observed variables in the whole research area [8]. Moran's I measures the relationship between spatial elements, which is similar to the correlation coefficient in statistics. Its value ranges from −1 to 1. If it is greater than zero, it indicates a positive correlation; if it is less than zero, it indicates a negative correlation; if it is equal to zero, it indicates no spatial correlation [9]. Moran's I index is greatly influenced by the spatial weight matrix, and the global space can explore the change rule of the spatial correlation of housing price under different spatial weights [10]. Significant Moran's I value indicates that the price of new residential buildings in urban areas has spatial agglomeration, that is, plots with high prices gather together, and plots with low prices gather together [11]. Luo and Wei analyzed the land value of Milwaukee by geostatistical method, and found that urban land price has significant spatial correlation, and there are differences among different locations and land use properties [12]. Liu et al. used the global autocorrelation model to find that China's real estate prices present a positive spatial correlation on the whole. For each region, the spatial spillover effect of real estate prices in the eastern and central regions is significant, and the real estate prices in the eastern region have a stronger spatial positive correlation [13].

Space Markov chain method is the traditional method of Markov chain and regional condition. Markov chain method optimized combination, giving full consideration to the space between the time series of regional interaction, through spatial weight matrix that can solve the problem of the spatial relations between areas, and with the aid of lagging behind the concept of space, define each field of spatial neighborhood. Thus, the spatial effects of geographical environment on regional development are quantitatively analyzed [14–17]. After analyzing the change of housing price in Britain, Sean Holly found that the change of housing price in London would lead to the change of housing price in other areas, and such influence had a certain lag [14]. Xue Liang used spatial Markov chain model to quantitatively study the ecological security and economic level of Guanzhong region and summarized its spatial-temporal evolution characteristics [15, 18]. Zhou Li used traditional Markov chain and spatial Markov chain methods to construct nonspatial and spatial Markov transfer probability matrices of rural economic development level, respectively, and analyzed and predicted the evolution characteristics of spatial-temporal pattern of rural economic development level in the research period [16]. Yan Tao et al. used spatial data statistical analysis model and spatial Markov model to analyze regional differences and spatiotemporal evolution characteristics of Urban economic development in China from 2001 to 2016 [17].

## 3. Data Sources and Research Methods

### 3.1. Data Sources

Four districts, one city, and four counties are under the jurisdiction of Hefei city. This paper mainly selects four municipal districts of Hefei (Yaohai district, Luyang District, Shushan District and Baohe District) as the research scope (As shown in Figure 2), and collects the price data of 353 second-hand housing in Hefei from 2020 to 2021. Among them, the sample panel data comes from Anjuke, and the spatial vector data of the base map comes from the national basic data of the National geographic Information Resource Catalogue Service system, through the use of Baidu map to pick up and edit coordinate information, combined with ArcGIS, GeoDa, and Matlab software for data processing and analysis.

### 3.2. Research Methods

#### 3.2.1. Spatial Autocorrelation

(1) Global autocorrelation model. Global autocorrelation is used to quantitatively describe the average degree of association of all spatial units with neighboring regions over the whole region, so as to determine whether the phenomenon exists in spatial agglomeration. In this paper, Global Moran's I is selected to reflect the overall distribution of commodity housing prices in each neighborhood, and its calculation formula is as follows.
  (1) Global Moran's I=n∑i=1n∑j=1nWijyi−y¯yj−y¯∑i=1n∑j=1nWij∑i=1nWijyi−y¯2,
where *y*_*i*_*y*_*j*_ is the house price of the ith and jth cell, respectively, $\bar{y}$ is the mean value of house prices of all cells, *W*_*ij*_ is the value of spatial weights between cell *i* and cell *j* (the spatial weight matrix of distances is constructed in this paper), and *n* is the total number of cells studied.
(2) Local autocorrelation model. Local autocorrelation can be used to reflect the degree of spatial correlation between local study units in the study area and the values of similar attributes in the surrounding area, and the calculation formula is
  (2) Local Moran's I=nyi−y¯∑j=1mWijyi−y¯∑i=1nyi−y¯2,
where *y*_i_ is the house price of the ith, W_ij_ is the spatial weight value between cell *i* and cell *j*, n is the total number of cells studied, and *m* is the number of cells adjacent to cell *i*.

#### 3.2.2. Kriging Interpolation Method

The Kriging interpolation method is a method for unbiased optimal estimation of regionalized variables within a certain region based on the theory of variance function and structural analysis [6, 7]. The Kriging interpolation method considers the correlation between cells, and the test results are more informative in the case of multiple sample points. In this paper, the general kriging interpolation method, which has a wide range of applications, is used to interpolate housing prices, and its formula is as follows:

(3) $$\begin{array}{c} \overset{\wedge }{Ζ}\left(x_{0}\right)=\sum_{i=1}^{n}\lambda_{i}Ζ\left(x_{i}\right). \end{array}$$

$\overset{\wedge }{Z}$ (*x*_0_) denotes the predicted value of the unknown point, Z(*x*_i_) denotes the value of the surrounding known points, *λ*_i_ denotes the weight of the ith known point on the unknown point, and *n* is the amount of sample data.

#### 3.2.3. Markov Chain

Markov chain is a stochastic process in which both time and state are in a discrete state. In the process of analysis, continuous values are discretized and divided into *k* types by numerical rank, and then the probability distribution of each type and its interannual variation are calculated to approximate the evolution of things. The expressions are as follows:

(4) $$\begin{array}{c} {\text{m}}_{ij}=\frac{n_{ij}}{n_{i}}, \end{array}$$

where *n*_*i*_ is the number of dwellings belonging to type *i* in the study time period, and n_ij_ refers to the number of residential buildings that changed from type *i* in *t* years to type *j* in *t* + 1 years during the study period.

#### 3.2.4. Spatial Markov Chain

Traditional Markov chain can count the spatiotemporal evolution of second-hand housing prices, unable to analyze the influence of the economic development in the region of neighborhood region, and thus on the basis of traditional Markov chain, it is introduced into the spatial lag conditions to build the space of the Markov chain, which is an effective analysis of the regional economic development and its surrounding residential environment for residential type change in the price. The spatial lag operator corresponding to the spatial lag operator is often used in spatial autocorrelation analysis. The spatial lag of a local area is the weighted average value of the observation values around the location; that is, the product (*WX*) of the regional observation vector (*X*) and the spatial weight matrix (*W*) is used to determine the neighborhood state of the region. It provides a method basis for quantitative analysis of regional spatial distribution pattern [17].

(5) $$\begin{array}{c} L\text{ag}=\sum_{i=1}^{n}x_{\text{i}}w_{ij}, \end{array}$$

where Lag is the spatial lag operator, *x*_*i*_ is the attribute value of the regional cell, and *w*_*ij*_ is the weight of the observation of domain *j* for the spatial lag operator at location *i*. The traditional *k* × *k* Markov matrix is decomposed into *k* × *k* × *k* conditional transfer probability matrices conditional on the spatial lag according to the economic state or type of the adjacent region. *m*_*ij*_ (*k*) denotes a spatial transfer probability conditional on the spatial lag type of the cell at moment *t*, which is transferred from type *i* to type *j*. By comparing the traditional Markov matrix with the spatial Markov transfer matrix to explore the probability of upward or downward transferring of a study unit, the transformation of different used residential price types in different neighborhood environments can be analyzed, and the degree of influence of the neighborhood environment on the price transfer of used residential units can be studied.

## 4. Empirical Analysis

### 4.1. Spatially Divergent Characteristics of Second-Hand House Prices in Hefei City

#### 4.1.1. Global Autocorrelation

In this paper, the global Moran's I index of second-hand residential prices in Hefei city from 2020 to 2021 are calculated based on the spatial weight matrix of Euclidean distance (Table 1).It can be seen from the table that all the global Moran's I indices are positive, and are between 0.6037 and 0.6896, with a confidence of 99%. The results show that the second-hand houses in Hefei urban area have significant spatial correlation effect and show agglomeration phenomenon in space. Among them, under the influence of the new real estate policy, Moran's I index of second-hand housing price in Hefei decreased from 0.6883 to 0.6791 in a short period after April. It shows that the agglomeration effect is slightly weakened, and the trend of housing price growth has been temporarily controlled.

#### 4.1.2. Local Autocorrelation

The global Moran's I index shows that there are different levels of spatial clustering of second-hand residential prices in Hefei city, which does not show the spatial clustering characteristics of second-hand residential prices in Hefei city. Therefore, this paper adopts the LISA diagram of local autocorrelation to analyze the spatial distribution and spatial clustering characteristics of residential prices in Hefei city.  Figure 3 shows the spatial agglomeration of housing prices in the four phases.

As shown in Figure 3, the “high-high” agglomeration is mainly distributed in the area of Shushan District, such as the governmental affairs district board, Huang Qianwang board, Economic Development District board, and Binhu New District board. The “low-low” agglomeration is mainly distributed in the northeastern area, such as Yaohai Old Town board, Xinzhan District board, and partial Luyang District board. The residential houses in the “low-high” agglomeration are mainly scattered around the “high-high” agglomeration, and the number is gradually decreasing, while the residential houses in the “high-low” agglomeration are more spatially dispersed, and the number of “high-low” clusters is spatially dispersed and remains low for a long time.

Figure 3(a) shows: in October 2020, “high-high” concentrated in the government affairs area of Shushan District, closely surrounding Swan Lake and municipal government affairs center, such as The Arch of Triumph, Ink Orchid Pavilion, Swan Lake bank and Sansheng Yi Garden. “Low-low” residential cluster is mainly distributed in Yaohai district and Yaohai district and Luyang district junction; “high-low” cluster houses are small in number and scattered around “low-low” cluster houses, located at the intersection of Luyang and Yaohai old city; “low-high” clustered houses are mainly distributed around “high-high” clustered houses, between government district and economic district, and the rest are scattered in Huangqianwang plate.

Figure 3(b) shows the following: compared with October 2020, in January 2021, “high-high” clustered residences are still mainly concentrated in the government affairs district board and Binhu New District board in Shushan District, among which Binhu New District expands 5 “high-high” clustered objects; the number of “low-low” clustered residences increases, mainly in Baohe District, and the location north of the junction of Luyang District and Yaohai District; “high-low” clustered and “low-high” clustered residences do not change significantly in spatial location, and increase or decrease in quantity.

Figure 3(c) shows that, compared to January 2021, the “high-high” agglomeration in April of that year expanded in the governmental district section of Shushan District and the Binhu New District section, and the degree of expansion was not obvious; the distribution pattern of the “low-low” agglomeration changed more, except for the local areas along the Banqiao River in Yaohai District and Luyang District, and the increase in the number in Baohe District was more obvious, mainly in the location north of Taihu Road, such as Chengjian Century Garden and the Youth District. The “high-low” agglomeration and the “low-high” agglomeration do not have significant changes in the space and number of residences.

Figure 3(d) shows, that compared with April 2021, the location of “high-high” agglomeration in July of that year has not changed significantly, but the number of “high-high” agglomeration has increased slightly compared with the previous one, mainly in Baohe District, such as Edinburgh of World Jincheng, Windsor City of World Jincheng and Oriental Residence in Baohe District; the number of residences in “low-low” agglomeration has decreased in Baohe District, but they are still concentrated in Yaohai District and its surroundings; “high-low” agglomeration is scattered around the residences in “low-low” agglomeration and the number has decreased. There is no significant change in the number of “low-high” clusters, and only one place in Shushan District, Newspaper Park (East), is influenced by the surrounding “high-high” clusters to change from “low-high” clusters to “high-high” clusters.

### 4.2. Overall Divergent Characteristics of Second-Hand House Prices in Hefei City

#### 4.2.1. Kriging Interpolation Method

The Kriging interpolation analysis method using the spatial distribution tool of ArcGIS was used to locally interpolate the residential price data to generate a continuous price surface, as shown in Figure 4.

According to the results of Kriging interpolation analysis, the housing prices in hefei urban area decrease from west to east and from south to north, which can be summarized as the distribution of “two points and one side”. Two “points” are Shushan district and Binhu New District, which are two areas with high housing prices, while “one side” is Luyang District and Yaohai District, which are relatively low and evenly distributed. At the same time, the areas with high housing prices gradually decrease from the circle to the periphery and the grading is obvious. There is no obvious leap-over phenomenon, and the housing prices show a certain agglomeration phenomenon in the region. Since the implementation of the New Deal, Yaohai district and its surrounding old city in the long-term low value level, only a few local areas of the price growth trend. There may be several reasons for the long-term low value of Yaohai District and its surroundings:

1. Luyang District and Yaohai District, as the old urban areas of Hefei, carry the history of urban development, and their old planning and old buildings lead to land scarcity to limit their real estate development potential.
2. For a long time, Luyang district and Yaohai District have been the economic center and industrial center of Hefei respectively. The government and enterprises have built low-income housing such as demolition houses and public rental houses to solve the housing problem of the working population. As a result, residents in the old city have no more demand for housing.
3. The excessive development and use of the old city makes the blocks appear to be “old and small, dirty and messy,” but the poor living environment limits the rise of housing prices. From the point of view of spatial distribution, the local area of Baohe River region changed from high to low, and then remained stable. It shows that there is a certain “inflated price” problem in the reduced regional price, and the “inflated” regional price drops to the “real” level. Shushan district and Binhu New District have obviously slowed down the trend of outward diffusion, price growth has slowed down. This shows that housing prices in Shushan district and Binhu New Area have gradually returned to a state of stable growth after the impact of policy adjustment.

### 4.3. Time Evolution Characteristics of Second-Hand House Prices in Hefei City

#### 4.3.1. Markov Shift Matrix

With the support of ArcGIS software, the Markov shift probability matrix of the second-hand residential property prices in Hefei city was obtained by overlaying the data of previous years (as shown in Table 2).

1. As can be seen from Table 2, the larger values in the matrix of residential price types in the two different time periods are concentrated on the main diagonal, which indicates that the residential prices in the second-hand residential market in Hefei city have a high stability in the process of development. From the values on the diagonal, it can be seen that the probability of residential prices maintaining their original level type in the first six months is at least 88.9%, and the probability of residential price levels maintaining their original state in the second six months is at least 87.6%. Compared with the first six months, the ability of residential prices to maintain their original level in the later period affected by policy regulation has slightly decreased, and policy regulation has played a certain effect.
2. Different types of residential prices are affected by policy adjustments to different degrees. As can be seen from Table 2, the probability of low level, low and medium level, and high level types of residential to maintain their original state has decreased by the impact of policy regulation. Among them, the probability of upward shift of low and lower level increases, while the probability of upward shift of medium and high level types of residential houses decreases, and only the probability of maintaining their original level is high. This indicates that the medium and high level types of housing are more influenced by the policy, and the target of policy regulation is more clear.
3. Each stage still presents upward development trend. Overall, the probability sum of the upper triangle and the lower triangle in stage 1 is 0.205 and 0.065, respectively, and the probability sum of the upper triangle and the lower triangle in stage 2 is 0.205 and 0.064, respectively. The probability sum of the upper triangle of the two stages is larger than that of the lower triangle, which shows that the probability of upward transfer of the housing price type is larger than that of downward transfer, indicating that the housing price presents an upward development trend in general.
4. Most residential prices maintain their original state, and the lowest probability of maintaining their original level is 87.6%, which is higher than the probability of the price type shifting to other types. This indicates that there is a “club convergence” of residential price types, and most residential prices tend to converge to higher or high-economic types.

#### 4.3.2. Spatial Markov Transfer Matrix

The traditional Markov chain approach is based on the assumption that regions are independent of each other, thus ignoring the positive and negative influence of the neighborhood environment in the dynamic evolution of the region. Residential neighborhoods are relatively small regional units, but they do not exist independently, and they are interconnected with the surrounding areas. Therefore, based on the traditional Markov transfer probability matrix, the spatial Markov chain transfer probability matrix is constructed by introducing the condition of spatial lag through Matlab software (see Table 3).

1. Residential neighborhood background plays an important role in the development of residential economy. The probability of economic type transfer is different for a house in different neighborhood. If a house is adjacent to a house with a low price level, it will be negatively affected by the neighborhood, resulting in a negative spatial spillover effect and difficult to move up. When it is adjacent to the house with a higher price level, the positive spillover effect will be generated, which inhibits its downward transfer and promotes its upward transfer. As a result, the house price gradually tends to the same level in space, which provides a spatial explanation for the phenomenon of “club convergence.”
2. Different neighborhood environments play different roles in the process of residential price shift. For example, the probability of upward shift is 0.041 and downward shift is 0.020 when a higher type residential neighborhood is adjacent to a lower type residential neighborhood in Stage 2, and 0.178 and 0.000 when it is adjacent to a high type residential neighborhood. 13.7 percentage points, while its probability of downward shift decreases by 20 percentage points. This indicates that the probability of upward shift increases when a residential neighborhood is adjacent to more developed residential houses; on the contrary, the probability of upward shift is suppressed when it is adjacent to less developed residential houses.
3. Policy adjustments play different roles for different types of residences. As a result of the policy, the upward shift of low and low-middle level types of residences is promoted, while the shift of middle and high level types of residences is suppressed. For example, the probability of upward shift for low and medium level types of dwellings in the same medium and high level neighborhood environment is 0.074 for Stage 1 and 0.129 for Stage 2, representing a 5.5% increase in the probability of upward shift. The probability of upward shift of stage 1 to 0.064 and upward shift of stage 2 to 0.043 for the higher level type of housing in the high level neighborhood environment decreased by 2.1%.

## 5. Research Conclusion

This paper analyzes the spatiotemporal evolution characteristics of residential prices in Hefei city by using kriging interpolation, spatial autocorrelation, and spatial Markov chain, based on the study of 353 residential community price seats in Hefei city from 2020 to 2021. The following conclusions are drawn.

1. From the perspective of spatial pattern, the residential houses in Hefei city show the situation of “two points on one side,” the high level of residential prices is mainly concentrated in the south and southwest of Hefei city, while Yaohai district and its surroundings have been at low level for a long time, and the residential development is divided between north and south. Hefei city residential prices have obvious clustering phenomenon, HH clustering of residential drive obvious role.
2. From the perspective of time evolution, under the influence of different neighborhood environments, the neighborhood with higher price level will increase the probability of upward transfer and inhibit the possibility of downward transfer, and the spatial convergence of clubs is presented overall. At the same time, under the short-term influence of the policy, the housing prices of low level and middle and low level are promoted in the same neighborhood environment, while the housing prices of high level and middle and high level are negatively affected.
3. Generally speaking, the policy has a positive regulation effect on the housing price of high level and high level type and promotes the transfer of low level and low level price type. Limited by the “old broken small, dirty and messy” living environment and the scarcity of development resources, the housing price in the old city of Hefei has a slow growth, but compared with Shushan District, Binhu New Area and new station area, the housing price in the old city is still in the overall low value level for a long time, the growth power is insufficient. The government district and Binhu New Area, as new areas with policy-oriented resource input, always make clear the spatial layout of community living circle, gradually improve the future-oriented growth public service system, and provide public service guarantee for all ages, with strong community public service and green livable ability. As a result, housing prices have remained high for a long time.

## Figures and Tables

**Figure 1:** Organizational flow chart.

**Figure 2:** Distribution of Hefei city districts.

**Figure 3:** Local spatial distribution of second-hand residential prices in Hefei city, 2020–2021.

**Figure 4:** Distribution of kriging space of second-hand residential prices in Hefei city in April and September 2021.

**Table 1:** Global Moran index of second-hand residential prices in Hefei city, 2020–2021.

	Moran's I	*Z* score	*P* value
Oct.	0.6037	25.6593	<0.001
Nov.	0.6079	25.8290	<0.001
Dec.	0.6305	26.7703	<0.001
Jan.	0.6430	27.2898	<0.001
Feb.	0.6450	27.3593	<0.001
Mar.	0.6848	29.0196	<0.001
Apr.	0.6883	29.1532	<0.001
May.	0.6825	28.8979	<0.001
Jun.	0.6791	28.7499	<0.001
Jul.	0.6850	28.9959	<0.001
Aug.	0.6896	29.1880	<0.001
Sept.	0.6890	29.1619	<0.001

**Table 2:** Markov shift probability matrix of second-hand residential prices in Hefei city, 2020–2021

Local status	2020.10–2021.3 (stage 1)					2021.4–2021.9 (stage 2)				
	*n*	Low	Lower	Higher	High	*n*	Low	Lower	Higher	High
*t*/*t* + 1	1765	<25%	25%∼50%	50%∼75%	>75%	1765	<25%	25%∼50%	50%∼75%	>75%
Low	448	**0.946**	0.054	0.000	0.000	449	**0.931**	0.069	0.000	0.000
Lower	447	0.034	**0.897**	0.069	0.000	444	0.025	**0.876**	0.099	0.000
Higher	449	0.000	0.029	**0.889**	0.082	433	0.000	0.028	**0.935**	0.037
High	421	0.000	0.000	0.002	**0.998**	439	0.000	0.000	0.011	**0.989**

**Table 3:** Spatial Markov transition probability matrix of secondary residential prices in Hefei city in 2020–2021 (conditional on spatial lag).

Spatial lag	Local status	2020.10–2021.3 (stage 1)					2021.4–2021.9 (stage 2)				
		*n*	Low	Lower	Higher	High	*n*	Low	Lower	Higher	High
	*t*/*t* + 1	1765	<25%	25%∼50%	50%∼75%	>75%	1765	<25%	25%∼50%	50%∼75%	>75%
*Low*	Low	313	**0.968**	0.032	0.000	0.000	318	**0.950**	0.050	0.000	0.000
	Lower	75	0.080	**0.920**	0.000	0.000	59	0.102	**0.831**	0.068	0.000
	Higher	25	0.000	0.000	**1.000**	0.000	16	0.000	0.063	**0.938**	0.000
	High	0	0.000	0.000	0.000	0.000	0	0.000	0.000	0.000	**0.000**

*Lower*	Low	94	**0.904**	0.096	0.000	0.000	91	**0.890**	0.110	0.000	0.000
	Lower	97	0.052	**0.887**	0.062	0.000	166	0.012	**0.898**	0.090	0.000
	Higher	98	0.000	0.020	**0.939**	0.041	89	0.000	0.067	**0.921**	0.011
	High	5	0.000	0.000	0.000	**1.000**	8	0.000	0.000	0.000	**1.000**

*Higher*	Low	37	**0.865**	0.135	0.000	0.000	40	**0.875**	0.125	0.000	0.000
	Lower	230	0.017	**0.909**	0.074	0.000	194	0.015	**0.856**	0.129	0.000
	Higher	249	0.000	0.040	**0.896**	0.064	253	0.000	0.016	**0.941**	0.043
	High	89	0.000	0.000	0.011	**0.989**	103	0.000	0.0	0.019	**0.981**

*High*	Low	4	**1.000**	0.000	0.000	0.000	0.000	**0.000**	0.000	0.000	0.000
	Lower	45	0.000	**0.822**	0.178	0.000	25	0.000	**1.000**	0.000	0.000
	Higher	77	0.000	0.013	**0.766**	0.221	75	0.000	0.013	**0.933**	0.053
	High	327	0.000	0.000	0.000	**1.000**	328	0.000	0.000	0.009	**0.991**

## Data Availability

Sample data on second-hand home prices used to support the results of this study are included in the supplementary information document. These datasets were derived from the following public domain resources: https://hf.anjuke.com/sale/?from=navigationhttps://map.baidu.com/@13057397.574469628,3719598.6899990723,12.3z

## Supplementary Materials

Supplementary Materials Analyze data as attachment: Data.xlsx.(Supplementary Materials).
